This article has been retracted.

# Nervonic acid amends motor disorder in a mouse model of Parkinson’s disease

**DOI:** 10.1515/tnsci-2020-0171

**Published:** 2021-05-25

**Authors:** Dandong Hu, Yujuan Cui, Ji Zhang

**Affiliations:** School of Life Science, Northwest Normal University, Lanzhou, Gansu 730070, People’s Republic of China; Beijing Yanqing District Food and Drug Safety Monitoring Center, Beijing Yanqing Center for Diseases Prevention and Control, Beijing, 102100, People’s Republic of China

**Keywords:** Parkinson’s disease, nervonic acid, motor disorder

## Abstract

**Objectives:**

Parkinson’s disease (PD) is a kind of common neurodegenerative disease in the world. Previous studies have proved that nervonic acid (NA), extracted from *Xanthoceras sorbifolia* Bunge, has the potentials of neuroprotection. However, the effect of NA on the PD remained unknown. This study was designed to investigate the NA’s potential function and relative mechanism on motor disorder.

**Methods:**

1-Methyl-4-phenyl-1,2,3,6-tetrahydropyridine (MPTP) was used for producing parkinsonism motor disorder on male C57BL/6 mice. Toxicity experiments and behavioral assay were performed to evaluate the effect of NA. Besides, the expression levels of tyrosine hydroxylase and α-synuclein, as well as striatal dopamine (DA), serotonin, and their metabolites were explored through immunoblotting and chromatography after NA treatment *in vivo*.

**Results:**

We found that NA could alleviate the MPTP-induced behavioral deficits dose-dependently. Moreover, NA has no toxic effects on the mouse liver and kidney. Of note, we found that NA significantly reduced the impact of MPTP impairment and striatal DA, serotonin, and metabolites were remained unaffected. In addition, tyrosine hydroxylase was upregulated while α-synuclein being downregulated and the oxidative stress was partially repressed evidenced by the upregulation of superoxide dismutase and glutathione activity after NA treatment.

**Conclusion:**

Our findings unveil NA’s potential for protecting motor system against motor disorder in the PD mouse model without any side effects, indicating NA as an alternative strategy for PD symptom remission.

## 1 Introduction

Parkinson’s disease (PD), as the second grave health problem of neurodegenerative diseases, is affecting about 3% of the population aged over 60 [1]. With the growing number of the aging population, the incidence of PD grows substantially [2]. The typical symptom of PD is motor disorder, with muscle rigidity, bradykinesia, tremor, and postural instability [3], while other multiple non-motor symptoms include sensory, emotional, cognitive, and autonomic defects [4]. Intensive studies suggest that the procession, reduction in dopaminergic neurons in the substantia nigra pars compacta, and the accumulation of Lewy bodies in neurons, which are the basic pathologically features of PD, result in the motor symptom [5]. Therefore, the downregulation of dopamine (DA) in striatum and upregulation of α-synuclein are the hallmarks of PD. Nowadays, the development of serotonergic pathology is earlier than that of dopaminergic pathology during the formation of PD, especially in those who carry the specific α-synuclein mutation. Therefore, serotonin (5-HT) is highlighted to be a novel marker of PD [6]. Based on these mechanisms, several therapy strategies are investigated to alleviate or suppress this neurodegenerative disease, among which DA supplementation with drugs, including l-3,4-dihydroxyphenylalanine (l-DOPA), DA agonist, and monoamine oxidase B (MAO-B) inhibitors [7], is used to inhibit DA breakdown or activate DA receptor. However, these treatments may cause various severe side effects and drug resistance. Moreover, nondopaminergic therapies, such as inosine, iron chelators, and anti-inflammatories, as well as non-pharmacological approaches (e.g., gene therapies and neurotrophic factors) have been strongly supported by pre-clinic studies [8,9], while no approach has convincingly showed the advancement in the clinic. Therefore, it is of great essential to further investigate new therapeutic strategies for PD since its multiple clinical phenotypes.

Currently, some traditional Chinese medicine (TCM) has been applied for improving motor disorders in PD, including tremor and head-shaking [10]. The *Xanthoceras sorbifolia* Bunge, which is also denoted as a yellow horn in China, is an oil-rich seed shrub and possesses multiple pharmacological properties [11,12]. Of note, nervonic acid (NA) is the main active compound of this TCM. It is a kind of the primary long-chain fatty acids and has been reported to associate with the brain development and could attenuate various neurological diseases [13]. For instance, Amminger et al. found that NA is an essential constituent of myelin. Lack of NA may promote the conversion to psychosis in patients with prodromal symptoms [14]. Similarly, increased levels of plasma NA is a common trend in the major depressive disorder, bipolar disorder, and schizophrenia patients, indicating it was an available marker for diagnosis [15]. Vozella et al. found that age-dependent accumulation of NA-containing sphingolipids and NA-synthesizing enzyme is presented in the aged hippocampus, indicating these aggregations’ contribution to normal and pathological brain aging [16]. Thus, NA may have a preferable neuroprotective effect and could be considered as a supplement for PD treatment. Here, we construct the 1-methyl-4-phenyl-1,2,3,6-tetrahydropyridine (MPTP)-induced PD mice model for NA functional study. We presented that NA could reduce the motor deficits though increasing the levels of striatal DA, 5-HT, and TH, as well as decreasing the α-synuclein expression and oxidative stress, thereby providing further insights into novel candidate drug for PD therapy.

## 2 Materials and methods

### 2.1 Chemicals

NA (90%) was purchased from Hengke biotechnology Co. (Shanghai, China, CAS.No:506-37-6). The MPTP was purchased from Sigma (St. Louis, USA).

### 2.2 Animals

The male C57BL/6 mice (8–10 weeks old, 20–22 g) were purchased from Nanjing Medical University Animal Laboratory, housed in a standard animal house with free access to food and water. All animal treatment and behavioral assay were performed during the light cycle. To test the effects of NA alone on motor and biochemistry endpoints, 20 mice were randomly grouped into four groups (*n* = 5), including the control group, high dose group (60 mg/kg of NA), middle dose group (40 mg/kg of NA), and low dose group (20 mg/kg of NA). Except for the control group, the mice of other groups were treated by NA (*ig.*, 100 g of NA was mixed with 30 mL polysorbate-80, and then dissolved in PBS) at different concentrations for 10 days. Mice in the control group were treated by an equal volume of PBS. To determine the effects of NA against MPTP-induced toxicity, 25 mice were randomly divided into five groups (*n* = 5), including the control group, model group, high dose group (60 mg/kg of NA), middle dose group (40 mg/kg of NA), and low dose group (20 mg/kg of NA). Except for the control group, the mice of other groups were treated by MPTP (20 mg/kg, *i.p.*, dissolved in PBS) for the first 3 days to induce the experimental PD model. Then NA at different concentrations was treated by gavage (*ig.*). Mice in the control group and model group were treated by an equal volume of PBS. Further studies were performed 7 days later [17]. The control group was treated by vehicle without MPTP stimulation. The model mice were subjected to vehicle treatment after MPTP administration.


**Ethical approval:** Animal experiments are entirely in accordance with the guidelines of the National Institutes of Health, and the protocol used in this study was approved by the Committee of Northwest normal University.

### 2.3 Quantification of AST, ALT, superoxide dismutase (SOD), and glutathione (GSH)

The mice were anesthetized using isoflurane, while the brain was removed and washed by PBS for several times. The striatum was isolated and homogenized with 50 mM Tris HCl, pH 7.4 (1/10, w/v) immediately. Then the homogenate was centrifuged for 10 min at 10,000× *g*. The supernatants were used to test the level of SOD and GSH by the commercial kits (Jiancheng Bioengineering Institute, Nanjing) according to the manufacturer’s instructions. The mouse serum was collected to test the levels of glutamic-oxalacetic transaminase (AST) and glutamic-pyruvic transaminase (ALT) by the commercial kits (Jiancheng Bioengineering Institute, Nanjing) according to the manufacturer’s protocol.

### 2.4 Histological analysis

The mice were anesthetized 24 h after the last treatment. The liver and kidney tissues were isolated immediately. The tissues were then fixed with 4% paraformaldehyde for 48 h at 4°C. Subsequently, the tissues were embedded in paraffin and cut into 5 μm sections. Then the sections were stained by a hematoxylin and eosin staining kit (Abcam, China) following the manufacturer’s protocol. Finally, the sections were observed using a light microscope.

### 2.5 Behavioral testing

#### 2.5.1 Pole test

The test was performed based on previous studies [18,19]. In brief, a 9 mm diameter wooden pole was fixed in a cage. The mice were allowed to habituate to the environment at least 1 h before the test. The animals were placed on the top of the pole (length was 1 m) and faced upwards. The time of the animals took to descend to the ground was recorded.

#### 2.5.2 Rotarod assay

The rotarod test was used to evaluate the effect of NA on the mouse motor coordination and balance. The experiment was performed according to the previous studies [18,19]. In brief, mice were allowed to habituate to the environment at least 1 h before the test. Then, the mice were placed on an acceleration rod (4–40 rpm, for a maximum of 5 min). The latency for the first fall was recorded.

#### 2.5.3 Open field test

This experiment was performed as described earlier [20,21]. Briefly, mice were placed at the testing room to habituate to the environment before the test. For each test, animals were gently placed into the central area of a square wooden box (60 × 60 cm^2^). The movement and behavior were recorded using a Digiscan Monitor (Omnitech Electronics). Data were recorded at every 10 min interval. The wooden box was wiped by the ethanol solution and dried before the next test.

### 2.6 High-performance liquid chromatography (HPLC) analysis

The homogenate of the striatum was collected and centrifuged as described previously herein. The supernatant was collected to analyze the concentrations of striatal DA, 5-HT, and related metabolites (3,4-dihydroxypheny-lacetic acid [DOPAC], homovanillic acid [HVA], and 5-hydroxyindolacetic acid [5-HIAA]) using HPLC with electrochemical detection as described previously [22,23,24]. For DA and 5-HT, we used a mobile phase (75 mM sodium acetate, 15 μM EDTA [pH 6], 16% methanol, 3 mM sodium dodecylsulfate, and 16% acetonitrile). The mobile phase (100 mM KH_2_PO_4_, 10 mM sodium heptanesulfonate, 150 μM EDTA [pH 3.9], 5% methanol, and 5% acetonitrile) was used to analyze the metabolites. They were pumped at a flow rate of 0.5 mL/min on a C18 reversed-phase column (Agilent Technologies) and were quantified by an electrochemical analytical cell (CoulArray model 5600A). All data analysis was performed using CoulArray version 3.10 software (ESA Inc.).

### 2.7 Western blot assay

The striatum was isolated from the mice with different treatments. The tissues were then lysed by RIPA lysis buffer containing 1% PMSF and 1% protease inhibitor. The protein concentration of the total proteins was detected by a BCA protein kit (Sigma, USA) according to the manufacturer’s protocol. Equal amounts of proteins of each sample were loaded and separated by 10% SDS-PAGE, and transferred onto polyvinylidene difluoride membranes. After being blocked by a 5% non-fat milk solution for 1 h at room temperature, the membranes were incubated with primary antibodies overnight at 4°C. Subsequently, the membranes were washed and incubated with the second antibodies (anti-mouse IgG or anti-rabbit IgG, 1:10,000) for 2 h at room temperature. Finally, the membranes were imaged using an ECL kit (Thermo, USA) and quantified with Image J software. The primary antibodies against tyrosine hydroxylase (TH, 1:1,000), α-synuclein (1:1,000), and beta-actin (1:5,000) and secondary antibody (1:10,000) were purchased from Abcam (Shanghai, China).

### 2.8 Statistical analysis

Behavioral testing was performed at two different occasions. The data were analyzed by GraphPad Prism 7.0 (GraphPad, USA) and were shown as the mean ± SEM, *n* = 5, *p < 0.05, **p < 0.01, ***p < 0.001 vs the control group. ^#^ *p* < 0.05, ^##^ *p* < 0.01, ^###^ *p* < 0.001 vs model group. Differences between the selected groups were compared by one-way ANOVA, followed by Dunnett’s tests. A value of *p* < 0.05 was considered statistically significant for all analyses.

## 3 Results

### 3.1 Toxic effect of NA *in vivo*

We first detected serum levels of AST and ALT to evaluate the liver function in the male C57BL/6 mice. The results showed that the administration of NA at different doses alone presented no significant fluctuation on serum AST and ALT levels when compared to the controls (Figure 1a). To further evaluate the potential toxicity of NA to the liver, we analyzed liver histopathology features by H&E staining after NA treatment. As shown in Figure 1b, an abundant apparent nucleus and entire cytoplasm were presented in the control group. Moreover, the liver cells showed a mesh-like appearance with clear boundaries and arranged around the central vein. We found no statistical difference among NA treatment groups and the control group. Similarly, kidney tissues of the control group presented the typical appearance of the complete proximal convoluted tubule, and distal convoluted tubule structure, as well as clear cortical or medullary structures [25]. The images of different doses of treated mice appeared similar to the features as in the control group. Our results demonstrated that NA showed no toxic effects on the liver and kidney, even at the highest dose.

**Figure 1:** NA displayed no toxicity on mouse liver and kidney. (a) Mice were treated with indicated doses of NA; serum levels of AST and ALT were detected. (b) Representative H&E images of livers and kidneys from mice treated by NA at different concentrations.

### 3.2 NA reversed behavioral deficits in the PD mice model

Next, to find out the *bona fide* impact of NA on motor function, the mice were monitored by the pole test, rotarod assay, and open field test at day 7. In the pole climb assay, the climbing time was dramatically increased in the PD mouse model, with 34.7 ± 2.43 s in the model group and 6.32 ± 1.12 s in the control group (*p* < 0.01). However, the climbing time of the NA-treated mice was dramatically decreased in a NA dose-dependent manner (*p* < 0.05). Besides, the effect of NA on PD-induced behavioral deficits was also evaluated by the rotarod test. Compared with the control group, the mean time of rolling showed a 50% reduction in the MPTP-induced PD model. In contrast, NA treatment reversed this deficit at all evaluated doses (*p* < 0.05). For the open field evaluation, the number of spontaneous movements was significantly reduced after PD operation, with 68.59 ± 6.48 turns/min in the model group and 94.26 ± 9.17 turns/min in the control group (*p* < 0.05). In contrast, the NA administration showed a neuroprotective effect. The mice presented more spontaneous movements than the model group. The number of spontaneous movements increased from 75.61 ± 8.33 turns/min to 87.31 ± 7.8 turns/min. However, only those treated with a high dose of NA (>40 mg/kg) presented a significant difference compared to the model group (*p* < 0.05).

### 3.3 Effect of NA on DA, 5-HT, and their metabolites in the striatum

To investigate whether the NA administration protects against the degeneration of the dopaminergic system, we evaluated the concentration of DA, 5-HT, and related metabolites in striatum. MPTP treatment significantly declined the expression levels of striatal DA and related metabolites, including DOPAC and HVA. The levels of DA were decreased approximately five-folds as compared with that in the control group (*p* < 0.05) (Figure 2a–c). Compared with the model group, the mean concentration of DA and related metabolites was significantly increased in response to middle dose (40 mg/kg) and high doses (60 mg/kg) NA treatment. Consistently, similar trends were observed in the striatal 5-HT and related metabolite – 5-HIAA. In detail, the levels of 5-HT and 5-HIAA were decreased by about 70.2 and 71.4% in the model group, respectively, when compared with those in the control group. However, with the NA treatment, the levels of 5-HT and 5-HIAA were normalized dose-dependently (Figure 2d and e). All the aforementioned evidences indicated that NA prevented the loss of DA and 5-HT in the PD model. Moreover, we observed a marked reduction in striatal TH, which is a marker dopaminergic system, in the MPTP-induced mouse model (Figure 2f). In contrast, 40 and 60 mg/kg doses of NA treatment significantly increased the protein expression levels of TH (*p* < 0.05), while the low dose of NA treatment produced a gentle upregulation. The current results suggested that NA showed a protective effect on the dopaminergic system, which was in agreement with the results of the improvement of motor disorder (Table 1).

**Figure 2:** NA upregulated striatal DA, 5-HT, and their metabolites as well as TH of the MPTP-treated mice model. The level of DA (a), 5-HT (b), DOPAC (c), HVA (d), and 5-HIAA (e) in the striatum of mice with different treatments were detected by HPLC, respectively. (f) Change in TH protein level between different NA administration group was detected by western blot (left) and the relative quantification was calculated (right), which showed the protein expression levels of TH and β-actin of five groups and the quantitative analysis chart. Data were shown as the mean ± SEM. *N* = 5, *p < 0.05, **p < 0.01, ***p < 0.001 vs the control group. ^#^ *p* < 0.05, ^##^ *p* < 0.01, ^###^ *p* < 0.001 vs model group. The control group was treated by vehicle without MPTP stimulation. The model mice were subjected to vehicle treatment after MPTP administration.

**Table 1:** Effects of NA on motor activities of the MPTP-treated mice model

Group	Climbing time (s)	Rolling time (s)	Number of spontaneous movement
Control	6.32 ± 1.12	584.23 ± 18.37	94.26 ± 9.17
Model	34.7 ± 2.43^***^	241.38 ± 15.67^***^	68.59 ± 6.48^**^
NA (20 mg/kg)	15.56 ± 1.97^##^	317.26 ± 16.29^#^	75.61 ± 8.33^#^
NA (40 mg/kg)	12.61 ± 1.03^##^	354.71 ± 18.35^#^	83.26 ± 7.51^#^
NA (60 mg/kg)	9.84 ± 0.95^##^	410.3 ± 16.72^##^	87.31 ± 7.8^#^

The motor functions of mice were tested by pole test, rotarod assay, and open field test. The mean climbing time, rolling time, and the number of spontaneous movements were recorded. Data were shown as the mean ± SEM. *N* = 5, *p < 0.05, **p < 0.01, ***p < 0.001 vs the control group. ^#^ *p* < 0.05, ^##^ *p* < 0.01, ^###^ *p* < 0.001 vs model group. The control group was treated by vehicle without MPTP stimulation. The model mice were subjected to vehicle treatment after MPTP administration.

### 3.4 NA inhibited the α-synuclein expression and regulated oxidative stress response

We further investigated whether NA affected α-synuclein expression *in vivo*. MPTP treatment significantly upregulated α-synuclein expression in the striatum, whereas the NA reduced the expression of α-synuclein in a dose-dependent manner (*p* < 0.05) (Figure 3a). In addition, considering that the increased oxidative stress can cause α-synuclein aggregation, we detected the levels of the antioxidant markers (e.g., SOD, and GSH) in the striatum of mice. Compared with the control group, the MPTP-treated mice displayed lower SOD and GSH activity in the striatum. The activities of SOD and GSH were reduced to about 70 and 65% in the model group, respectively. However, NA significantly increased the activity of the SOD with 25% increase at a low dose, 50% increase at middle dose, and 51% increase at high dose. Besides, GSH protein level in the PD mouse model was also markedly improved by NA treatment, with 10% increase at a low dose, 55% increase at middle dose, and 60% increase at high dose, respectively (Figure 3b).

**Figure 3:** NA downregulated α-synuclein with an ameliorated oxidative stress on the expression of α-synuclein and oxidative stress. (a) Western blot analysis of the protein expression levels of α-synuclein and β-actin of five groups and the quantitative analysis chart. Change in α-synuclein protein level between different NA administration group was detected by western blot (left) and the relative quantification was calculated (right). (b and c) Activities of SOD and GSH in the striatum of mice with different treatments. Data were shown as the mean ± SEM. *N* = 5, *p < 0.05, **p < 0.01, ***p < 0.001 vs the control group. ^#^ *p* < 0.05, ^##^ *p* < 0.01, ^###^ *p* < 0.001 vs model group. The control group was treated by vehicle without MPTP stimulation. The model mice were subjected to vehicle treatment after MPTP administration.

## 4 Discussion

Currently, multiple animal models established on mice, rat, and non-human primate are being studied for the PD pathological process and the potential candidates’ evaluation [26,27]. As a kind of neurotoxic pollutants, MPTP is widely used to induce a PD-like pathology in rodent animals. Blood–brain barrier (BBB) could not intercept this neurotoxin. Once MPTP enters the brain microenvironment, it is metabolized into 1-methyl-4-phenylpyridinium (MPP^+^), which is toxic for nervous system [28]. MPP^+^ could be further transferred into dopaminergic neurons, leading to the loss of dopaminergic neurons or inhibiting mitochondrial function [29]. As a result, the oxidative stress response, mitochondrial dysfunction, and inflammation have been initiated, which are involved in the procession of PD [30]. What is more, except for the reductions of DA and TH, MPTP administration also causes behavioral deficits [31]. This model shows a high similarity with PD. In our study, the climbing time dramatically increased, while the mean time of rolling showed a significant reduction after MPTP treatment. Besides, the mice showed less spontaneous movements in the open area. Moreover, along with the downregulation of the striatal DA and TH, a high level of α-synuclein and low activation of oxidative stress were presented in our model. Therefore, we had successfully established a PD mice model with the motor deficits.

α-Synuclein, which is an important protein associated with PD, is significantly increased by MPTP and destroys the BBB in the substantia nigra pars compacta. Increased α-synuclein may activate glial cells to induce inflammation and in turn it also promotes its own expression. α-Synuclein dysfunction plays key roles in Parkinsonian degeneration leads to lose formation of myelin structure induced by MPTP indicates, PD degeneration is related to α-synuclein-induced myelin damage [32]. It is well known that NA is biosynthesized at the same time as myelinogenesis occurs and plays an important role in forming the plasma membrane’s lipid bilayer and in maintaining normal myelin function. Literature suggests a high expression of synuclein MPTP-induced injury. In light of the synuclein alterations, it can be suggested that, and by targeting this protein, one may modulate MPTP neurotoxicity in PD [33]. Dysfunction of oligodendrocytes (OLs) is regarded as one of the major causes of inefficient remyelination in multiple sclerosis, but their physiological capability to myelin synthesis is limited. Study has revealed that during acute inflammation such as in an experimental autoimmune encephalomyelitis brain, lipid metabolism pathway shifts toward synthesis of common substrates into proinflammatory arachidonic acid production, and NA synthesis is silenced [34]. Thus, increased levels of plasma NA might reflect dysregulation of OLs, sphingomyelin-rich lipid rafts, and/or the sphingomyelin metabolic pathway in patients with MDD [15]. Lower essential lipids may account for increased demyelination and the reduced efficiency of the remyelination process. Kageyama et al. (2018) indicate that NA compound does not pass through the BBB [15]. Earlier published reports have stated putative mechanism for fatty acid transport into cells. One proposed mechanism states that fatty acid merely diffuses into the exofacial leaflet of the plasma membrane in response to flipping of cytofacial leaflet. Negative charge on the carboxylic acid presents a limiting factor in terms of thermodynamic challenge for cytofacial leaflet flipping [35].

In recent years, as a complementary strategy of pharmacological treatments, many natural products based on foods or plants have been used to treat multiple diseases [32]. The relevant compounds, which were extracted from 38 herbal medicines, such as *Acanthopanax*, *Alpinia*, and *Astragalus*, showed promising effects on PD [33]. In this study, we highlighted the *in vivo* pharmacologic effects of candidate compound – NA. Interestingly, NA has no toxic effect on liver and kidney, even with the highest dose (60 mg/kg) treatment, which was much higher than the recommended dose of the mainstream drugs [34,35]. Furthermore, we found that NA partially protected against MPTP-induced motor deficits and displayed a neuroprotective response in our PD model. Compared to our drug, some conventional drugs such as levodopa and lazabemide were found to increase adverse motor effects, including dyshinesia and motor fluctuation, and even notable mortality rate [36,37]. These results indicated that NA was a safe drug for PD treatment.

Given that DA, 5-HT, and α-synuclein were the hallmarks of PD [38,39], we further investigated whether NA could affect these molecules. As expected, administration of NA after MPTP treatment avoided the reduction of striatal DA, striatal 5-HT, as well as their metabolites content. In contrast, with the NA treatment, the reduction of striatal α-synuclein was seen. Moreover, NA treatment contributed to prompt the production of TH, which was a marker enzyme that indirectly influences the activity of central DA neurons [40,41]. We further confirmed that NA could ameliorate oxidative burden of PD mice striatum by the upregulated activity of anti-oxidative enzyme, which are SOD and GSH in this paper, leading to the loss of α-synuclein. Blocking DA metabolism or activating DA receptors can regulate the movement ability of organisms [7]. These findings suggested that NA may be a novel effective medicine for PD. In summary, our findings demonstrated that NA possessed neuroprotection abilities against PD via the regulation of the dopaminergic system and the suppression of oxidative stress, thus ameliorating motor disorder of PD mice.
